# Method, Design, and Evaluation of an Exoskeleton for Lifting a Load In Situ

**DOI:** 10.1155/2021/5513013

**Published:** 2021-05-25

**Authors:** Xin Li, Weihao Li, Qiang Li

**Affiliations:** School of Mechanical and Materials Engineering, North China University of Technology, Beijing 100144, China

## Abstract

Due to the unclear application scenarios and force analysis of exoskeletons, there exists a research gap in exoskeleton design. This paper presents a design method and realization of an exoskeleton for a specific scenario of lifting a load in situ. Firstly, the lifting motion process and its data were collected based on a 3-D motion capture system and dynamometer treadmill system. Then, the variations of the torque and motion of each joint were obtained from the data analysis, based on which an active assistance mode for upper limbs and a passive assistance mode for lower limbs were demonstrated. In this design, the hydraulic cylinder for shoulder assistance, the motor for elbow assistance, and the spring for lower limb assistance were calculated and selected according to the motion and torque of each joint. Finally, subjective and objective methods were used to evaluate the exoskeleton based on the results of five test participants, and the median oxygen consumption of the whole test by lifting a load ten times with the assistance was found to be reduced by 9.45% as compared with that in the absence of the exoskeleton.

## 1. Introduction

The rapid development of internet technology has not only introduced convenience to daily life but has also promoted the expansion of the logistics industry. Robots have been applied in some logistics tasks, such as handling, grabbing, and placing items with regular shapes; however, robots cannot replace human beings for the handling of goods with uncertain shapes, sizes, or weights. There are nearly 50 million logistics employees in China, and many (<40 years old) who work under high-intensity conditions without limb protection have suffered from tenosynovitis, lumbar disc herniation, or other diseases. Therefore, it is necessary to provide protection to ensure the health of the limbs and joints of these workers.

An exoskeleton is a functional device that attaches to the human body to assist specific joints to protect or strengthen the body. According to the different application scenarios of products, the modes of exoskeletons can be generally categorized into rehabilitation [1–5], industry [6], and military [7] applications; for industry and military applications in particular, the exoskeleton supplements normal human power to conduct lifting. Generally, active assistance and passive assistance [8] are two common driving modes, and active assistance modes can be further divided into hydraulic [9], motor-driven [10, 11], and pneumatic [12, 13] modes. The power systems of hydraulic or pneumatic driving modes introduce additional load to the body due to their large volume; in contrast, a motor can be placed on the back of the body. Among the limb assistance components, assistance for upper limbs (shoulder [14], elbow [15], and wrist [16] joints), the waist joint [17], and lower limbs (hip [18], knee [19], and ankle [20] joints) has been developed. Moreover, some exoskeletons, called exosuit, have no rigid frame [21]. An exosuit is driven by a motor and a Bowden cable that is fixed on the end of the motor, and force can be transferred to any limb joints by the Bowden cable [22]. From the perspective of control methods, electromyography (EMG) signals [23] or end force/torque detection [24] are usually regarded as the control input. Regarding exoskeleton evaluation, the subjective feeling of wearers and the results of an objective test have been illustrated to evaluate a passive exoskeleton [25].

As is evident from the preceding review, there are numerous structural, driving, and control modes that can be adopted in exoskeleton design. However, exoskeletons are not generalized devices; the ignorance of the influence of the working scenario or working load on human limbs will lead to the inapplicability of exoskeleton design. For example, rehabilitation exoskeletons are usually oriented to patients with physical disabilities, who rely on the exoskeleton to provide fixed movements to perform rehabilitation and physical therapy on the limbs. Therefore, the emphasis of rehabilitation exoskeletons is usually placed on the movement of specific joints. The portability of wear and weight are two aspects of exoskeleton product. In contrast, for industrial or logistics applications, the target is normal people with a certain labor intensity. In this case, comfortable wear is almost as important as the effectiveness of assistance; otherwise, unfriendly human-exoskeleton interaction would directly affect the wearer's work efficiency. Moreover, the design of exoskeletons requires analysis to determine which joints or limbs require assistance based on the application scenario, which has been omitted in traditional research.

There has been less research on exoskeletons for use in industry or logistics applications than on exoskeletons for use in rehabilitation. Li et al. [26] presented an active dual-arm exoskeleton that can be adapted to various environments by adjusting the force and impedance adaptation, such as lifting loads or rehabilitation training. Yu et al. [27] illustrated an upper-limb exoskeleton for refractory construction, which can be used to reduce the physical fatigue of operators resulting from long hours of working with heavy loads; however, this active exoskeleton has the deficiencies of a greater self-weight and unfitness for walking. Koopman et al. [28] presented a light and convenient exoskeleton for lumbar protection in logistics work. Dinh et al. [21] illustrated an exosuit that reduces the muscular effort required to lift 1 kg by 48.3%. Picchiotti et al. [17] compared two commercially available postural assist exoskeletons and reported that there is no significant biomechanical benefit regarding the joint flexion angles and moment arms for lifting a given load. As is evident, although passive exoskeletons or exosuits are characterized by improved human-machine interaction, they are not suitable for large loads. Consequently, it is important to consider the application scenario and human-machine interaction as the design bases.

This study presents a complete method of exoskeleton design that is oriented to packing and lifting in logistics work. The remainder of this research is organized as follows.  Section 2 presents the design and analysis process of the exoskeleton under the suggested scenario.  Section 3 illustrates the motion capture and data analysis regarding the movement of entire limbs, based on which the kinematics and torque of joints are obtained.  Section 4 reports the calculation and design of the exoskeleton, which consists of elbow, shoulder, and lower limb assistance, as well as an electrical system.  Section 5 illustrates the prototype and experiments, the results of which verify the effectiveness of the design process.

## 2. Exoskeleton Design and Analysis Process

As mentioned in the previous section, exoskeletons are not universal products; thus, the working environment, the wearer's motion, and the assistance performance must be included as design inputs. The design and analysis process is illustrated in Figure 1.

According to the figure, the design process of the exoskeleton can be divided into the following five steps: the input of the working condition, motion capture, data analysis, system design, and test evaluation. First, the input of the working condition requires the analysis of exoskeleton application scenarios, such as the working environment, load profile, and human characteristics, based on which misunderstandings of exoskeleton design can be avoided. Second, the torque and motion of the joints should be tested based on 3-D motion capture equipment, from which the values of the torques, angles, and muscle activity of human limbs can be obtained. Third, the joint torque data can guide the maximum capacity and selection of joints for exoskeleton design, and the data of joint motion can be used to determine the speed and motion range of limbs. Fourth, the energy and drive systems are designed based on the joint torque data and assistance efficiency. Additionally, the structure and mechanical system are designed based on the joint motion data. Then, the exoskeleton prototype system is assembled based on the structure and electrical system. Finally, the results of objective tests and subjective feelings about the exoskeleton prototype can be evaluated. In particular, the assistance efficiency of the prototype should be compared to the design values, based on which the system design can be optimized.

## 3. Motion Capture and Data Analysis of Lifting Load In Situ

### 3.1. Experimental Scenario

The scenario considered in this research was a logistics sorting operator lifting a load from the ground to a certain height in a fixed operation area. The load mass was set as 20 kg, and the lifting heights were, respectively, set as 1 m and 1.5 m. To obtain clear and complete data on the lifting process, a 3-D motion capture system (Phasespace, Impulse X2E) was adopted to collect data on the lifting movement of the whole body and each joint; 36 marker points were stuck on the body of the wearer, and 10 cameras captured the motion. Additionally, a dynamometer treadmill system (Bertec FIT, FITITC-11-20L) was used to obtain the plantar force (see Figures 2 and 3). Then, OpenSim (V4.0) software was used to collect data on the motion and plantar force, based on which the motion of the limbs and the torque of the joints of the test participants were obtained.

### 3.2. Analysis of Experimental Data

Figure 3 depicts the experimental scenario of the lifting test. Data were collected from the 3-D motion capture system and dynamometer treadmill system to determine the motion of the limbs and the torque of the joints of the participant, after which the data were imported into OpenSim software to restore the participant's motion and determine the motion variation process, as shown in Figure 4. This process was primarily conducted to verify the effectiveness of the data collection of the 3-D motion capture system and to provide support for the inverse kinematics solution of the torques of the joints in the subsequent step.

Figure 5 reveals the height variation of the lifted load collected by the 3-D motion capture system, which meets the design requirements.  Figure 6 presents the variations of the angles of the hip, knee, ankle, shoulder, and elbow joints in the extension/flexion degree of freedom (DOF) when lifting the load. The first lifting phase was from the ground to a height of 1 m, and the second lifting phase was from the height of 1 m to the height of 1.5 m. As shown in Figure 6, during the first lifting phase, the lower limbs of the participant gradually changed from the bending state to the upright state; specifically, the hip joint changed from 90° to -10°, the knee joint changed from -130° to 0°, and the ankle joint changed from 32° to -7°. During the second lifting phase, there was almost no change in any joint of the lower limbs. Regarding the upper limbs, the angle of the shoulder joint was 90° when the participant grabbed the load on the ground; it was reduced to 50° after the first lifting phase, and it finally increased to 75° during the second lifting phase. The angle of the elbow joint changed little during the first lifting phase and increased from 10° to 55° during the second lifting phase. Additionally, the rotational speeds of the limb joints were obtained based on Figure 6. In the first lifting phase, the average speeds of the hip, knee, and ankle joints were found to be 75°/s, 76.47°/s, and 18.82°/s, respectively. Regarding the upper limbs, the rotational speeds of the elbow and shoulder joints in the second lifting phase presented faster variations than in the first lifting phase, and the maximum rotational speeds were about 40.9°/s and 41.7°/s, respectively. These kinematic values of the limbs and joints provide the basis of the structural and system design of the exoskeleton system.

As lifting in situ is primarily completed in the sagittal plane, the extension/flexion DOF of each joint provides more support for lifting. As shown in Figure 7, the torque value of the flexion DOF was much higher than that of the side-up and rotation DOFs. Therefore, this paper focuses on the analysis of the extension/flexion DOF of each joint.

Figure 8 presents the torque variations of the hip, knee, ankle, shoulder, and elbow joints in the extension/flexion DOF during the lifting process. The torque amplitudes of the joints in the lower limb were found to be higher than those of the joints in the upper limb. In addition, the torque values of the upper-limb joints are positive because the rotational direction of torque acting on the elbow and shoulder is clockwise; specifically, the latissimus dorsi behind the shoulder is mainly responsible for its flexion, and the bicipital muscle on the upper limb is mainly responsible for elbow flexion. Regarding the lower limbs, the direction of DOFs of the hip and ankle joints is extension during the entire lifting process, and the direction of torque driven by the corresponding muscle to the joint is counterclockwise; thus, the values of their torques are negative. Regarding the knee, torque assists the extension DOF of the joint in the first lifting phase, the direction of which is clockwise, so the value is positive. Subsequently, the value changes to a negative value because the direction of DOF changes to flexion, which changes the direction of the joint torque to counterclockwise.

Regarding the torque amplitude, the value of the hip joint ranged from -95 to -70 Nm, that of the knee joint changed from 40 to -70 Nm, and that of the ankle joint ranged from -45 to -10 Nm throughout the entire lifting phase. During the first lifting phase, the torque of the shoulder joint was found to increase from 17 to 30 Nm, and that of the elbow joint increased from 0 to 10 Nm. During the second lifting phase, the torque of the shoulder joint was found to continually increase from 30 Nm to nearly 50 Nm, while the torque of the elbow joint increased from 10 to 18 Nm and then decreased gradually after reaching the peak; this occurred because the load was closer to the participant, and the load on the elbow joint gradually decreased while the angle of the shoulder joint increased.

According to the analysis of the motion and torque data of the joints of the participant, the following can be concluded: (1) the kinematic angle variations of joints can be used as the basis for the calculation of the extension value of the actuator of the exoskeleton assistance system; (2) the rotational speed of joints represents the basic movement speed of the actuator; (3) the motion and torque data of joints can be used as the basis for the selection of the energy power of the exoskeleton assistance system; and (4) the torque and motion of the joints of the upper and lower limbs can be used as the basis for the design of the exoskeleton structure and assistance mode. The next section describes the design of the exoskeleton system based on the preceding analysis.

## 4. Exoskeleton System Design

According to the kinematics and analysis of the joint torques in specific scenarios presented in the previous section, the exoskeleton assistance mode, structure of the limbs and joints, and corresponding electrical system are designed in this section.

### 4.1. Exoskeleton Assisting Mode

According to the torque data of each joint obtained in Section 3, the torque amplitude of each joint in the lower limb is higher than that of each joint in the upper limb. Moreover, there exist significant differences in the muscle groups that drive each joint [29, 30], and the volume of lower limbs is much larger than that of the upper limbs. Considering that the ankle joint bears a small torque when lifting a load, this paper focuses only on the analysis of the shoulder, elbow, hip, and knee joints.

The average muscle volume that drives each joint of the lower limb is significantly higher than that which drives each joint in the upper limb. Additionally, due to the gravity of the upper body, the flexion DOF of the joints in the lower limbs was found to require relatively less effort than the extension DOF when the participant tried to squat, so the lower limbs of the exoskeleton can be designed as passive spring assistance equipment. Consequently, the lower limbs must overcome the tension of a certain spring, which can also be used as the preload when lifting the load. In contrast, the upper limbs must provide active assistance due to the smaller muscle volume and heavy load imposed on the upper limbs.

From the perspective of the assistance mode, the upper limb has 7 DOFs. Previous studies [31, 32] usually tried to set the number of DOFs in the upper limb as high as possible, which would not only increase the mass of the exoskeleton but also introduce difficulty to posture detection and control; moreover, this makes it difficult to guarantee the effectiveness of the assistance of the exoskeleton. Therefore, in this study, the assistance mode was designed for the specific scenario of lifting a load in situ. Based on the data analysis conducted in the previous section, the forces on the shoulder and elbow joints are mainly focused on the flexion DOF; therefore, the assistance of the exoskeleton should also be emphasized for the flexion DOF. Additionally, due to the lifting of the load in situ, the driving energy system of the exoskeleton can be fixed outside the wearer's body, which could reduce the burden caused by the weight of the energy system. According to the preceding analysis, the design of the exoskeleton is illustrated in Figure 9.

As can be seen from Figure 9, the lower limb of the exoskeleton was designed as passive spring assistance. The spring is connected to the hip and knee joints by Bowden lines, which can flexibly transfer the force. Additionally, the springs extend when the wearer squats to grab the load, which provides the preload for the extension of the hip and knee. The elbow joint is assisted by a motor-driven Bowden line, and the shoulder joint is assisted by a hydraulic cylinder that pushes the upper arm. There are 2 DOFs with the upper limbs, and the advantage of this structure mode is that it avoids the complicated DOF fitting for the shoulder joint, and the energy system is set outside the body. The specific process of the lifting action is presented in Figure 10.

It can be seen from Figures 10(a) and 10(b) that when the wearer squats and starts to lift the load, the joints of the lower limbs are in a flexion state, and the hip and knee joints must overcome the tension of the spring, which is fixed at the back of the wearer. Additionally, the shoulder joint is also in a flexion state to grab the load, and the hydraulic cylinder then needs to be extended to support the upper arm. As shown in Figures 10(b) and 10(c), the spring preload acting on the hip and knee joints transforms the power to joint extension and assists the wearer to complete the upright action. Figures 10(c) and 10(d) reveal that the lower limbs remain upright, and the elbow and shoulder joints begin to flex with assistance from the motor-driven Bowden line and the hydraulic cylinder-driven hydraulic energy system, respectively, thereby completing the entire lifting movement process.

The following sections provide the details of the design and parameter calculation based on the assistance mode and motion data of each joint.

### 4.2. Design of Elbow Joint Assistance

Based on the physical measurements of the participants, the length of the upper arm was set as Ls = 350 mm and the length of the forearm was set as Lq = 400 mm. The other parameters were set according to the anchor position of the Bowden line on the upper limb, namely, L1 = 100 mm, L2 = 200 mm, L3 = 150 mm, L4 = 150 mm, and L5 = 80 mm.

The motor parameters were obtained based on the structure mode and force analysis. According to Figure 6, the angle and torque of the elbow joint changed little in the first lifting phase; however, in the second lifting phase, the angle of the elbow joint increased from 10° to 55°, and the torque power of the elbow joint also increased from 10 to 18 Nm. Thus, the maximum torque of the elbow joint was calculated according to the second lifting phase. The calculation of elbow joint assistance is based on Figure 11 (in which all the symbols are defined), as follows:

(1) $$\begin{array}{c} \omega_{1}=\text{arctg}\left(\text{L}5∕\text{L}4\right). \end{array}$$

According to Equation (1) and L3 = L4, the following can be calculated:

(2) $$\begin{array}{c} \omega =\beta /2+\omega_{1}. \end{array}$$

Then, the assisting torque *M*_*z*_ acting on the elbow joint by Bowden line is calculated as follows:

(3) $$\begin{array}{c} M_{z}=F_{z}\cdot \cos\omega \cdot \sqrt{\text{L}4^{2}+\text{L}5^{2}}. \end{array}$$

The load torque *M*_L_ acting on elbow joint is defined as follows:

(4) $$\begin{array}{c} M_{\text{L}}=G\cdot \text{Lq}\cdot \sin\left(\alpha +\beta \right). \end{array}$$

The tension force *F*_*z*_ of the Bowden line while in static or in slow motion can be calculated based on Equation (3) and Equation (4).

In this study, the load was set as 20 kg, and the transmission efficiency *η* of the motor–reducer–rotor–Bowden line system shown in Figure 12 was set as 60%. The radius *r* of the rotor is 50 mm. Therefore, the output torque *M*_G_ at the end of the reducer for one arm is given by Equation (5), and the variation process is presented in Figure 13.

According to Figure 6, the time of the 2^nd^ lifting phase was from 2.1 s to 3.8 s (the participant was in a static state after 3.8 s), which consisted of elbow flexion (2.1~3.2 s) and shoulder flexion (3.2~3.8 s). Moreover, the use of simultaneous elbow and shoulder flexion is simulated in Figure 13. We set course (*A*) as from position (*c*)~(*c*′)~(*d*), and course (*B*) as from position (*c*)~(*d*), which are shown as Figure 13.

(5) $$\begin{array}{c} M_{\text{G}}=\frac{0.5\cdot G\cdot \text{Lq}\cdot \sin\left(\alpha +\beta \right)\cdot r}{\cos\omega \cdot \sqrt{\text{L}4^{2}+\text{L}5^{2}}\cdot \eta }. \end{array}$$

Figure 13 exhibits the calculation results of the output torque with different flexion courses. In course (*A*), the maximum torque was found to be 33 Nm when the angle of elbow flexion increased to 55°, which was larger than that of course (*B*). However, the maximum torque required by the motor-reducer was considered as 33 Nm. Additionally, the maximum rotational speed of the elbow joint was found to be 40.9°/s, as calculated in Section 3.2. The linear velocity of the wire rope in the Bowden line should therefore be greater than 86.4 mm/s, so its rotational speed should be no less than 0.28 r/s. According to the torque and speed calculations, a MAXON servo motor RE65 was selected as the motor for elbow joint assistance, a GP81A model was selected as the reducer, and a Decathlon wire (diameter: 1.5 mm) was selected as the Bowden wire.

### 4.3. Design of Shoulder Joint Assistance

The shoulder joint is promoted by hydraulic cylinders. The pressure of the hydraulic energy system was selected as 16 MPa. Therefore, the size and stroke of the hydraulic cylinder were calculated and selected as follows based on the kinematics and dynamics of the upper limb. According to the initial state of the hydraulic cylinder shown in Figure 11, the distance between the two fulcrums is calculated as follows:

(6) $$\begin{array}{c} \text{Lyd}=\sqrt{\text{L}1^{2}+\text{L}2^{2}}=\sqrt{100^{2}+200^{2}=}223.6\left(\text{mm}\right). \end{array}$$

When the wearer squats and starts to lift the load, the hydraulic cylinder has the largest elongation, and the distance between the two fulcrums is as follows:

(7) $$\begin{array}{c} \text{Lyc}=\sqrt{{\left(\text{Ls}-\text{L}2+\text{L}1\right)}^{2}+\text{L}{\text{s}}^{2}}=\sqrt{250^{2}+350^{2}=}430.1\left(\text{mm}\right). \end{array}$$

Therefore, it can be concluded that the extension of the hydraulic cylinder should be at least 206.5 mm.

The distance from the lower fulcrum of the hydraulic cylinder to the shoulder joint Lp is as follows:

(8) $$\begin{array}{c} \text{Lp}=\sqrt{\text{L}1^{2}+\text{L}{\text{s}}^{2}}=\sqrt{100^{2}+350^{2}=}364\left(\text{mm}\right). \end{array}$$

According to the second lifting phase, some parameters are defined as follows:

- The arm of load L7 and the arm of assisting force L8 are as follows:

(9) $$\begin{array}{c} \text{L}7=\text{Ls}\cdot \sin\alpha +\text{Lq}\cdot \sin\left(\alpha +\beta \right),\\ \text{L}8=\left(\text{Ls}-\text{L}2\right)\cdot \sin\alpha \end{array}$$

(ii) The length Ly of the hydraulic cylinder in the second lifting phase is as follows:

(10) $$\begin{array}{c} \text{Ly}=\sqrt{{\left(\text{Ls}-\text{L}2\right)}^{2}+\text{L}{\text{p}}^{2}-2\left(\text{Ls}-\text{L}2\right)\cdot \text{Lp}\cdot \cos\left(\alpha +\gamma \right)} \end{array}$$

(iii) The angle  *δ* between the upper arm and the upper fulcrum of the hydraulic cylinder is as follows:

(11) $$\begin{array}{c} \delta =\arccos\frac{{\left(\text{Ls}-\text{L}2\right)}^{2}+\text{L}{\text{y}}^{2}-\text{L}{\text{p}}^{2}}{2\cdot \text{Ly}\cdot \left(\text{Ls}-\text{L}2\right)} \end{array}$$

According to Figure 14, the angle *δ* declines from 89.8° to 67° in the second lifting phase, which is the basis for the calculation of the force of the hydraulic cylinder.

(iv) Hydraulic cylinder output:

The working efficiency *ζ* of the hydraulic system was set as 50%, and the output force *F* of the hydraulic cylinder for one arm was calculated according to Figures 11(c) and 11(d), as follows:

(12) $$\begin{array}{c} F=\frac{0.5∙G\cdot \text{L}7}{\zeta ∙\text{L}8\cdot \sin\left(\delta -\left(\pi ∕2-\alpha \right)\right)}. \end{array}$$

If the pressure *P* of the hydraulic system is 16 MPa, the calculation of the inner diameter *d* of the hydraulic cylinder is as follows:

(13) $$\begin{array}{c} d=2\;\sqrt{\frac{F}{P\cdot \pi }}. \end{array}$$

Two different lifting courses were also calculated. The maximum force of the hydraulic cylinder occurred during elbow flexion in course (*A*), and its maximum value was larger than that of course (*B*). After calculation and comparison based on Figure 15, the diameter of the piston of the hydraulic cylinder should not be less than 10.9 mm, and 12 mm was selected for the design. Additionally, the maximum rotational speed of the shoulder joint was found to be 41.7°/s, as calculated in Section 3.2. The linear velocity of the hydraulic cylinder should therefore be greater than 106.7 mm/s. Then, based on the extension speed of the hydraulic cylinder and the diameter of its piston, the flow should not be less than 0.72 L/min. Consequently, the design of the hydraulic system can be obtained according to the calculation.

### 4.4. Design of Lower Limb Assistance

According to the structure mode presented in Section 4.1, the passive assistance mode was adopted for the hip and knee joints, for which the spring and wire rope in series were primarily used for assistance. As shown in Figure 16, one side of each wire rope was fixed on the hip and knee joints, respectively, and the other side was connected to the springs by pulleys. According to Figure 8, the maximum overcoming torques of the hip and knee joints in the first assisting phase are close to 95 Nm and 40 Nm, respectively. The parameters of the springs selected for the hip and knee joints are reported in Table 1, and the springs could, respectively, provide 796 N and 280 N of force for the extension of the joints. In addition, the maximum forces transferred by the Bowden lines to the hip and knee joints are, respectively, 47.76 Nm and 19.6 Nm, leading to a passive assistance efficiency of close to 50%.

### 4.5. Design of Electrical System

The electrical system of the exoskeleton includes a sensor unit, core processing unit, and execution unit. Among them, the sensor unit is mainly composed of internal measurement units (IMUs) and encoders. The IMUs are arranged along the sagittal plane of the thigh and calf. The encoders are placed at the hip joint and knee joint. The IMUs and encoders are primarily used to judge the posture of the lower limbs, which provides the control criterion for upper limb assistance. An NI sbRIO-9651 core processing unit was adopted as the bottom unit for data acquisition and information processing, and LabVIEW software was selected as the development environment of the upper computer. The execution unit was mainly divided into two parts, namely, the motor-driven Bowden line for the assistance of the elbow joint and the hydraulic cylinder-driven upper arm for the assistance of the shoulder joint. A MAXON EPOS4 50/15 module was adopted for the motor driver, while MAXON RE65 + GP81A modules were adopted for the motor + reducer. A small hydraulic station (16 MPa + 1 L/min) was adopted for the hydraulic system. The specific system composition is illustrated in Figure 17.

## 5. Test and Evaluation of Exoskeleton

### 5.1. Prototype Wearing of Exoskeleton

Based on the design, calculation, and model selection of the exoskeleton system described in the previous section, a prototype of the exoskeleton was assembled, as depicted in Figure 18. The prototype can be adapted to wearers with heights of 170-185 cm by adjusting the lengths of the upper and lower limbs. Moreover, the weight of the exoskeleton is only 6.8 kg, as the energy supply of the prototype is fixed outside the body. Additionally, the shoulder-assisting device driven by a hydraulic cylinder is placed on the back of the upper arm; thus, there is no interference with the shoulder movements, and the human-exoskeleton interaction is friendlier.

Regarding the control of the prototype, as the lower limbs are driven by passive power, the posture control strategy of the upper limbs can also be provided by IMU detection due to the movement relevance of the upper and lower limbs in the first lifting phase. In the second lifting phase, the upper limbs are driven by a motor + Bowden line and a hydraulic cylinder based on the position control. For the control of different lifting heights, the control parameters must be updated according to the actual scenario requirements.

### 5.2. Test Evaluation of Exoskeleton

A test evaluation of the exoskeleton system was carried out to verify its effectiveness and consisted of both objective evaluation and subjective assessment. Regarding objective evaluations, generally, the EMG signals of test participants wearing an exoskeleton system for single-joint assistance are collected and are then converted into muscle activation information as the evaluation criterion. Instead, aiming at exoskeleton systems for whole-body assistance, oxygen consumption data are collected and are characterized by comprehensive and objective evaluation. Therefore, in the present study, the oxygen consumption of the test participants was adopted as the objective evaluation criterion. Regarding subjective assessments, participants are usually asked to fill out questionnaires; this method was also adopted in the present study.

This study was approved by the Ethics Committee of North China University of Technology. The participants signed an informed consent form to participate in the study. The information about the five participants is reported in Table 2. Regarding the evaluation protocol, five participants each lifted a 15 kg load 10 times from the ground to a height of 1.5 m both with and without the exoskeleton, and a respirometer (COSMED K5) was used to record their oxygen consumption during each lifting of the load. Additionally, the quiescent oxygen consumption condition of each participant was collected. Then, the differences in the oxygen consumption during the lifting mode and quiescent condition were obtained and were employed as the objective evaluation data. For subjective assessment, each participant filled out a questionnaire at the end of the test to provide their subjective impression of the exoskeleton from five aspects, namely, perceived usefulness (PU, 0~10), side effect (SE, -10~0), intention of use (IU, 0~10), perceived ease of use (PEU, 0~10), and facilitating condition (FC, 0~10).  Table 3 shows the mean values and minimum values of the five participants' questionnaires.

The oxygen consumption of the five participants with and without the exoskeleton is presented in Figure 19. The median value of oxygen consumption was found to decrease by 11.3%, 6.79%, 6.28%, 10.4%, 11.26%, and 13.86% of five participants wearing exoskeletons, respectively. Regarding the values for the entire experiment, the median value of total oxygen consumption of five participants with exoskeletons reduced by 9.45% as compared with the absence of the exoskeleton, which demonstrates its assistance effectiveness. Moreover, as reported in Table 3, the five participants provided subjective evaluations of the exoskeleton from the aspects of PU, SE, IU, PEU, and FC, and the results indicate that the participants found the system helpful for decreasing physical fatigue. While no participant expressed any fear or concern about wearing the exoskeleton, the score of FC was lower than the scores of other aspects because the prototype is slightly difficult to wear and take off. Consequently, both objective evaluation and subjective assessment verified the effectiveness of the exoskeleton.

## 6. Conclusions

This paper presented the complete methodology, design, and test evaluation of an exoskeleton for use in the scenario of lifting a load in situ. The findings of the investigation can be summarized as follows:

1. The motion and torque of joints were analysed based on data collected from a 3-D motion capture system and dynamometer treadmill system. The rotational scope, speed, and torque of the joints when lifting a load in the sagittal plane were obtained and used as the basis for the system design of an exoskeleton
2. Based on the motion of the joints and a muscle layout analysis, an exoskeleton for use when lifting a load in situ was designed as including active assistance for upper limbs and passive assistance for lower limbs. Regarding the assistance of upper limbs, the energy system was designed to be placed outside the body, and the assistance mode of the hydraulic cylinder avoids interference between the exoskeleton and the body
3. Both objective and subjective methods were adopted for the evaluation of the designed exoskeleton. The median value of oxygen consumed by lifting a load ten times with the assistance of the exoskeleton was found to be reduced by 9.45% as compared with that in the absence of the exoskeleton. Additionally, the subjective feelings of test participants regarding the exoskeleton also proved its effectiveness

In future research, more details regarding the use scenarios of the exoskeleton will be included to design a structure and energy system, and the assistance efficiency will be promoted via the optimization of human-exoskeleton interaction.

## Figures and Tables

**Figure 1:** The design and analysis process of an exoskeleton.

**Figure 2:** Schematic diagram of the lifting test.

**Figure 3:** Experiment of lifting test.

**Figure 4:** The motion animation of the participant restored by OpenSim software.

**Figure 5:** The height variation of the lifted load.

**Figure 6:** Variations of joints' angles during lifting.

**Figure 7:** Torque variations of the three DOFs of the shoulder joint.

**Figure 8:** Torque variations of each joint during lifting.

**Figure 9:** Exoskeleton structure design. 1, upper arm bandage. 2, Bowden line connector of the elbow joint. 3, Bowden line wire rope of the elbow joint. 4, Bowden line anchor of the elbow joint. 5, forearm bandage. 6, Bowden line sheath of the knee joint. 7, Bowden line wire rope of the knee joint. 8, Bowden line anchor of the knee joint. 9, Bowden line sheath of the elbow joint. 10, motor system of the elbow joint. 11, hydraulic cylinder. 12, hydraulic pipe. 13, hydraulic energy system. 14, waist fixation block. 15, Bowden line wire rope of the hip joint. 16, Bowden line anchor of the hip joint. 17, exoskeleton frame. 18, spring for the knee joint. 19, pulley. 20, spring for the hip joint.

**Figure 10:** The process of lifting a load: (a) initial state; (b) squatting state; (c) lifting load to the upright position; (d) lifting the load to the target position.

**Figure 11:** Force analysis of upper limb movement: (a) initial state; (b) squatting state; (c) lifting load to the upright position; (d) lifting load to the target position state.

**Figure 12:** Schematic illustration of Bowden line driven by motor.

**Figure 13:** Torque variation at the end of the retarder with different flexion courses. Course (*A*) represents sequential elbow flexion and shoulder flexion. Course (*B*) represents simultaneous elbow flexion and shoulder flexion.

**Figure 14:** Variation of angle *δ*.

**Figure 15:** Variation of parameter *d* with different flexion courses.

**Figure 16:** The mode of lower limb assistance.

**Figure 17:** Schematic diagram of the exoskeleton electrical system.

**Figure 18:** Exoskeleton prototype: (a) profile of exoskeleton prototype; (b) adjustment of upper limbs; (c) adjustment of lower limbs.

**Figure 19:** Oxygen consumption of five participants.

**Table 1:** Selection of springs for the hip and knee joints.

Parameter	Knee spring	Hip spring
Spring material	SUS304	SUS304
Spring diameter (mm)	15	15
Spring wire diameter (mm)	3	4
Total laps	20	20
Initial length (mm)	80	100
Last length (mm)	100	120

**Table 2:** The information about the five participants.

Participant	Age	Height (mm)	Weight (kg)
P1	32	175	65
P2	36	185	80
P3	28	182	78
P4	24	177	75
P5	30	176	75

**Table 3:** Subject scores of the exoskeleton.

	PU	SE	IU	PEU	FC	Total
Mean	7.2	-3.1	8.1	8.3	6.5	27
Minimum	5.5	-5	7.5	7	5.5	20.5

## Data Availability

The data used to support the findings of this study are available from the corresponding author upon request.
